# Development and Optimization of Network Music Course Resources Based on Data Mining Technology under the Personalized Online Education Environment

**DOI:** 10.1155/2022/2876063

**Published:** 2022-09-26

**Authors:** Xiuli Yan

**Affiliations:** College of Music and Dance, Fuyang Normal University, Fuyang, Anhui 236041, China

## Abstract

The ever-evolving Internet technology has brought more information resources for music teaching than ever before. For music educators, figuring out how to create and use these tools more effectively has become a pressing concern. China will usher in a new age of innovation and integration between the Internet and different traditional businesses with the idea of “Internet Plus.” MOOCs present significant challenges to traditional teachers and teaching methods as a typical practice of the transformation of education informatization to innovation, and they also drive global education toward a new process of informatization development. This paper adopts Internet thinking as the guiding ideology for the development of future music education concepts and, concurrently, conducts specific transformation research based on Internet technology from four aspects: music teaching content, music teaching methods, music education concepts, and the passing down of traditional music culture. The improved association rule algorithm is used to organise the students' access data, decide which high-frequency websites are accessible to the students, and realize the intuitive positioning of high-frequency access and learning issues. Assist the school's decision-making and educational levels in identifying the issues that students have with their learning, and then, improve the network teaching platform's material to complete the task of personalized network education.

## 1. Introduction

In recent years, the development of computer software technology has changed people's work and life patterns. In terms of teaching, the way people acquire knowledge is also undergoing great changes. The situation of the original single mode of traditional education in the classroom is changing [1]. In the 1980s, information technology was gradually introduced into teaching, among which multimedia computer technology and network communication technology were the most representative [2].

Information technology is receiving more and more attention in education as it matures. “It offers a material and technological assurance for the coordination and collaboration of home education, social education, and school education, and it also provides significant support for the development of an overall and comprehensive education concept and education system” [3]. It engages students with a range of media content, creating a sound structure for the teaching process and producing the best possible learning outcomes. The practice of carrying out instructional activities utilizing multimedia computers and ready-made multimedia teaching software is now referred to as multimedia teaching [4]. However, there are also some issues with the study of music at the university level. For example, the influence of the examination-oriented education concept prevents students from developing their aesthetic education and overall quality, and there is no effective guarantee for the number of hours spent in class [5]. In addition, the dearth of teaching and educational resources is another crucial issue. The term “teaching resources” refers to the tools that teachers can use to implement the curriculum, which serves as the basis for all teaching activities. The effectiveness of educational activities is directly influenced by the structured and perfect nature of the educational resources [6]. For a long time, school resources have been the only resources in primary school music education. Specifically, they include primary school teachers, school teaching equipment, and teaching materials; with the continuous deepening of teaching practice, the limitations of school resources have become increasingly prominent. Weak teachers and single teaching materials have become the main factors restricting the teaching effect [7].

There are many different types of music curricular resources, and the extensive Internet platform offers a wealth of useful materials for their integration [8]. The network resources for music education span a variety of subject areas, demonstrating not only the depth and breadth of the network's resources but also their capacity to disseminate cutting-edge musical ideas, methods, and cultural advancements [9]. Considering the overarching objective of the current state of the Chinese school music curriculum, actively utilize the benefits of internet music resources to logically integrate and distribute teaching tools for music. Its ultimate objective is to improve the school music curriculum, the artistic lives of the students, their practice skills, their ability to think creatively, and the development of their self-control and sentiment. It is obvious that the broad network of music resources has significantly altered traditional music education and improved its connotation. Activities involving music education in schools have helped to organise curriculum and advance teaching methods. In order to promote the creation of online music education resources, it is imperative for music educators in the information age to integrate the emerging trend of information technology [10].

The primary objective of this study is to design and develop a music network teaching system based on the Moodle platform, integrate the teaching of the music subject with the teaching platform against the backdrop of current network technology, and achieve the networking of the teaching of conventional subjects using current technical means. The music course material is created using constructivism theory as a guide. Based on the core capabilities of the Moodle network platform, secondary development is done to expand the new learning activity function module to accommodate music teaching requirements and advance the system's effective design. The following are its innovations: (1) integrate the network-based teaching platform Moodle with the teaching of music; (2) implement the specific design of the music curriculum in the system, using constructivism theory as the guiding basis for curriculum development and design; and (3) redevelop the test plug-ins and homework plug-ins in the Moodle platform to meet the unique needs of the music courses in the system.

## 2. Related Work

China's data mining (DM) started relatively late, and it was also the first enterprise to develop in the early stage. However, at present, DM has not been accepted by the majority of users in China, and its utilization rate is not high, mainly because of security and other issues. However, domestic DM is developing rapidly, and all major enterprises, communication operators, and governments have established or are establishing data centers, with private cloud accounting for a large proportion. However, I believe that in the near future, the service model of DM will be accepted by the majority of users and then enter the mature stage of development.

Tsai and Wang designed a learning system using DM in the paper “Design of Lifelong Education Service Platform Based on Data Mining.” The system has flexible expansion ability and can be expanded at any time according to the needs of users [11]. Zhang made a preliminary study on the platform construction strategy of DM platform used in high education services and pointed out that DM plays a very important role in the informatization of high education. The author made a preliminary inquiry into how to build a DM platform in the field of education and, based on this, put forward the basic framework of the platform construction and made a comparative analysis of the modes of government and education departments participating in the construction [12]. He pointed out that the following measures can be taken to promote the development of DM in education: developing new applications based on DM, migrating users' information assets, building an “ecosystem” of education cloud, etc. A feasible direction for the future development of higher education cloud platform is pointed out [13]. Burak put forward that Internet thinking is not the exclusive thing of the Internet, nor an appendage that must be attached to Internet enterprises. It is a thinking mode that has been strengthened in all walks of life in recent years due to the vigorous development of the Internet age [14]. Asai and Yokoyama's research discusses how to apply the technological advantages of the new era to traditional music teaching, but it still does not extend the research perspective to the transformation of music education concept [15]. Xia and Xu proposed that the future music education must establish a national music education system. In the development of national music, we should not only pay attention to its historical position in China's development but should also integrate with the world's multiethnic music system to form national music that belongs to the new era and can be based in the world [16]. Huang and Wang believe that tapping the potential value of teaching materials and creating curriculum resources can promote the transformation of teaching methods and realize the effective utilization of resources. However, the application of teaching methods depends to a great extent on the present situation of their courses, because without their teaching materials and corresponding auxiliary materials, teachers will become “cooking without rice,” and their teaching will be impossible [17]. Yan thinks that to strengthen the guidance of learning style and cultivate students' ability to think independently and find and deal with problems, teachers must teach students to learn, reduce their dependence on teachers, and make them gradually have self-learning ability. At the same time, they should pay attention to students' individual development and cultivate their sense of participation [18]. In the article “Analysis of the Role of MOOC in Promoting the Balanced Develop of Piano Education in the East and the West,” Li focused on the analysis that the implementation of MOOC education in the western region will promote the piano education in the region and discussed the problems that need to be solved in the implementation of piano MOOC education [19]. Xia and Yan think that the above textbooks are not very suitable for freshmen and sophomores majoring in music. English auxiliary materials are also quite limited. All the English textbooks listed above have corresponding workbooks and CD-ROMs, whose purpose is to consolidate what we have learned. But students simply do not make full use of these resources. In addition, the leaders do not pay enough attention to the cultural knowledge of music majors, especially their English level, and their work focuses on mastering the professional knowledge of music students [20].

## 3. Methodology

### 3.1. The Idea of Online Music Education under the Internet Thinking

With the rapid development of computer industry and information science in the 21st century, the Internet has penetrated into every corner of people's lives all over the world, profoundly affecting the economic development of our society and people's lifestyle and quietly changing our thinking mode. Internet thinking refers to a commercial consciousness and idea with the color of the times, which is driven by electronic information technology and then formed in a special commercial environment. Generally speaking, Internet thinking is an inertia thinking mode formed with the rise of the Internet, which is generally more closely related to business. It can be said that it is an advanced business consciousness and idea that came into being in its special environment due to the entry of the Internet era. The core support of this thinking mode is the powerful database behind it. The traditional industry is bound to be greatly impacted by the Internet. This requires our traditional industry to keep pace with the times, use the spear of the other and attack the shield of the other, use this new Internet thinking to deal with the impact brought by information technology, and reexamine the market, users, and ecosystem. Music teaching system is to provide a centralized learning platform for students and teachers. Through this platform, teachers can release some teaching resources and make some learning plans. Students can immersively participate in the whole learning, download online, browse learning resources, and complete various learning tasks. In addition, there is no relevant supervision and supervision during online learning, so their enthusiasm is not high and the learning effect is not ideal.

The development of teaching strategies that reflect the fundamental ideas of the new curriculum is thriving under the direction of the new curriculum concept, and modern teaching is emerging on its own. The traditional emphasis on knowledge transfer in education has given way to a focus on student development in modern classrooms. Students are no longer passive recipients of information; the focus has shifted from a one-dimensional goal of emphasising knowledge and skills to one that encompasses emotions, attitudes, and values in a three-dimensional harmonious unity; and the relationship between teachers and students is one of student teacher and teacher student. Focus on developing students' practical skills and innovative spirit; switch from a single outdated teaching strategy to a more contemporary one with an innovation-focused approach. Although the music programmes at regional and national universities are more advanced educationally, they are fundamentally still a component of the teaching system and must prioritise enhancing the effectiveness and calibre of instruction. It is undeniable that the faculty members in the music departments of nearby universities, whether they are professors, associate professors, or lecturers, have unmatched advantages in terms of their knowledge of music theory, level of artistic ability, and capacity for conducting scientific research in the field of music. However, many teachers have glaring weaknesses when it comes to their actual teaching methods. It is not unusual for the classroom to be uninteresting and the instruction to be subpar, as shown in Figure 1.

MOOC is different from the previous network video open class or distance education. It consists of three parts: course micro video, course test and evaluation, and teacher-student interaction.

### 3.2. Research on Music Teaching Resource Sharing Based on Data Mining

DM technology benefits from the development of the Internet. According to China Internet Information Center, the development of information technology has made the database supporting technology develop by leaps and bounds, and the data content in the database has also been used by all walks of life. However, because of the development of Internet technology, computer technology, information technology, and the number of users, the amount of data in the database increases exponentially, which makes it difficult for people to make effective use of such a huge amount of data, and the authenticity of data is also a problem. In addition, data types and data security are also key issues in database use. In order to satisfy people's utilization of huge technologies, DM technology was created. DM technology is essentially a type of technology that processes data from databases using statistics. Its fundamental objective is to display it as quantitative, readily available data through data regularisation. The DM technology utilized in many fields is frequently defined in a constrained manner. We believe that the DM technology, when viewed from a technical standpoint, may be described as follows: it is a technical means to utilize various rules for directed data processing in a huge number of fuzzy, unsettling, random, and defective data and to extract data or laws helpful for some laws. Classification and prediction technology, cluster analysis technology, and association analysis technology are three categories of DM technology.

With the development and rapid development of the Internet, the size of the data set is getting larger and larger, so that there are Pb level data. Such massive data has exceeded the storage capacity of an independent physical computer. Therefore, it is necessary to partition such large-scale data set and then store the separated data on many independent physical computers. HDFS is a distributed file system with improved association rule algorithm, which is called improved association rule algorithm distributed file system. In informal documents or old documents and configuration files, it is sometimes referred to as DFS for short. HDFS, as a kind of “disk” for storing data, also has the concept of data block. However, the block of HDFS is a large data block of 64 MB by default, which can minimize the addressing overhead. Therefore, the files stored on HDFS will be divided into multiple blocks with set block size, and the blocks are independent of each other. However, unlike the previous file system, files smaller than one block size only occupy part of the space of the block. The reliability of HDFS files is because all data blocks will have copies when they are written into the file system. Generally, the default copy coefficient of data blocks is 3. The size of data blocks and the number of copies can be reconfigured. The file storage in HDFS is divided into many blocks with a specified data block size. The strategy of HDFS is to store these blocks in different datanodes as widely as possible. For example, when the client requests to write a file, the datanode directly responds to the request of the client and writes the file into the data block. When the client wants to query a file, the namenode responds. First, it needs to get the location list of the files requested by the client scattered in each datanode. After knowing that the files are stored on those datanodes, the client can directly read the files from the datanode. Based on the improved differential evolution clustering algorithm, collaborative filtering is performed to form a recommendation system, as shown in Figure 2.

Data reflects the law, and the law guides teaching. This concept is one of the core concepts of using big data to guide education and teaching. Modern education researchers explore the internal laws among the variables of education participants by developing DM models in different fields of education and refine the laws to provide feedback guidance, so as to facilitate the education decision-making level to plan and predict the overall trend and develop prospects of education. For example, there are great differences in education development, big data talents, and economic development among provinces in China. There is a gap in funding for the construction of the education big data platform. The big data application in the period of education transformation and development has low matching.

### 3.3. Algorithm Model Based on Improved Association Rules

Hadoop has its own distributed system, HDFS, whose full name is Hadoop Distributed File System. From the user's point of view, association rule is an important content in data mining, and it is also one of the first research contents. By using it, we can discover the relationships contained in data. The purpose of association rules is to find all concurrent relationships in data items, which are also called associations. It can be used to find the correlation of different items in the same event. The task of association rule mining is to discover strong rules from a given database. Before processing, users generally need to set a minimum support and a minimum credibility. Finding strong rules is usually divided into two processes. The first step is to discover frequent itemsets. To find all frequent itemsets, users must set a minimum support degree and then judge whether the support degree is greater than the minimum support degree, and the items that meet the conditions can form frequent itemsets. The most basic condition for forming association rules is to find all frequent itemsets, which can first find all the largest itemsets and then generate association rules. The second step is to generate the required rules according to frequent itemsets. In each maximum project set, an appropriate minimum confidence level can be specified according to the needs of users, and then association rules with confidence level greater than the specified value can be generated, as shown in Table 1.

The core selection strategy of the original standard scoring simplification algorithm in the calculation process is to cross intermediate individuals in the original population and then use the greedy strategy to select the appropriate data population to enter the next round of screening the original population, which can be shown by the following formula:

(1) $$\begin{array}{c} X_{i}\left(g+1\right)=\left\{\begin{array}{c} U_{i}\left(g+1\right),\text{if }f\left[U_{i}\left(g+1\right)\leq f\left[X_{i}\left(g\right)\right]\right],\\ X_{i}\left(G\right),\text{other}. \end{array}\right. \end{array}$$

In the process of improvement, we mainly optimized the selection strategy. In the process of improvement, a total of 2*N* individuals in the original population *X*_*i*_*g* and population *U*_*i*_(*g* + 1) were rearranged according to their adaptability. After arrangement, only the first *N* individuals with the best adaptability were selected to form a new population *W*, and then, the new population *R* was obtained after another population mutation by using the above compilation operation. To a certain extent, this improvement can make the original population search after self-global fusion before global search and automatically mutate and screen to generate better population individuals, which effectively reduces the convergence speed of the previous algorithm, but the overall convergence speed is basically unchanged.

It is a commonly used analysis statistic in distance clustering analysis. For samples with *p* variables, *n* samples can be regarded as *p* points in *n*-dimensional space. Naturally, it is conceivable to measure the proximity between samples by the distance between points, and *d*_*ij*_ is often used to indicate the distance between the *i* sample and the first sample. Distance similarity refers to the degree of similarity between two objects by the distance between them. The distance between two samples is between 0⟶∞. The smaller the distance, the closer the two samples are. There are the following three common distance similarities in cluster analysis.

Block distance

(2) $$\begin{array}{c} D_{ij}=\overset{p}{\underset{k=1}{\sum }}\left|Xik-Xjk\right|. \end{array}$$

Euclidean distance

(3) $$\begin{array}{c} D_{ij}=\left[\overset{p}{\underset{k=1}{\sum }}\left(Xik-Xjk\right)2\right]\frac{1}{2}. \end{array}$$

Ming's distance

(4) $$\begin{array}{c} D_{ij}\left(q\right)=\left(\overset{p}{\underset{k=1}{\sum }}\left|Xik-Xjk\right|q\right)\frac{1}{q},q>0. \end{array}$$

Obviously, when *q* = 1, the Ming distance will become the block distance. When *q* = 2, the Ming distance will become the Euclidean distance. Therefore, the Euclidean distance and the block distance are actually special cases of the Ming distance. The smaller the distance between two objects, the more similar the two objects are. The larger the distance between two objects, the less similar the two objects are.

If a given probability distribution of *P* = (*p*_1_, *p*_2_, ⋯, *p*_*n*_) is defined, the amount of information transmitted by this distribution is called the center of *p*, that is,

(5) $$\begin{array}{c} I\left(P\right)=-\left(p_{1}*\log_{2}\left(p_{1}\right)+p_{2}*\log_{2}\left(p_{2}\right)+\cdots +p_{n}*\log_{2}\left(p_{n}\right)\right), \end{array}$$

(6) $$\begin{array}{c} \text{INFO}\left(X,T\right)=\overset{n}{\underset{i=1}{\sum }}\left|T_{i}\right|/\left|T\right|\times \text{INFO}\left(T_{i}\right). \end{array}$$

Define the gain Gain(*X*, *T*) as

(7) $$\begin{array}{c} \text{Gain}\left(X,T\right)=\text{Info}\left(T\right)-\text{Info}\left(X,T\right). \end{array}$$

That is, the definition of gain is the difference between two information quantities, one of which is the information quantity of an element to be determined in *T*, and the other is the information quantity of an element of the factory to be determined after the value of the attribute *X* has been obtained; that is, the information gain is related to the attribute.

(8) $$\begin{array}{c} \sup\text{port}\left(X\right)\text{: }\sup\text{port}\left(X\right)=\frac{\left|X\right|}{\left|D\right|}*100\%. \end{array}$$

An association rule is an implication in the form of *X*⇒*Y*, where *X* ⊂ *D*, *Y* ⊂ *D* is the prerequisite of the rule and *X*∩*Y* = *Φ*, *X* is the result of the rule *Y*.

The confidence of rule *X*⇒*Y* in the transaction set database *D* is the percentage of the transactions containing item *D* in *X* to the transactions containing both item and item in *D*.

(9) $$\begin{array}{c} \text{Confidence}\left(X\Rightarrow Y\right)=\frac{\sup\text{port}\left(X\cup Y\right)}{\sup\text{port}\left(X\right)}. \end{array}$$

## 4. Result Analysis and Discussion

At present, great progress has been made in the construction of network music education resources in China, which is shown in the following aspects: some national network music education resource stations are playing an increasingly important role in the music teaching of domestic primary and secondary schools and even universities. Some specialized regional network music education resource centers led by government education departments have been built one after another, which has played a good role in integrating the network music education resource banks of subordinate counties, cities, and schools. Network music education resource stations in some professional fields have sprung up and become “bridgeheads” to popularize music knowledge and singing skills in this field. In addition, some personalized online music resource pages or sites have sprung up in the form of music blogs and personal music websites, which have played a positive role in promoting the popularization of music knowledge and the improvement of public music appreciation. (1) Zhongyin online: Zhongyin online is a national online music education website for music grade examination and music university entrance examination candidates. It is mainly characterized by the construction of online music courses. At the same time, it publishes various kinds of music information based on grade examination and art examination and has the function of popularizing music knowledge at home and abroad. The music knowledge involved in the “music school” section covers almost all kinds of music knowledge from the west to the nation, from ancient times to the present. It also introduces a lot of singing and playing experience and music education experience, such as “listening to the ‘old opera bones' of Beijing opera to talk about the art of drama,” “basic practical knowledge of saxophone flute heads and whistles,” and “analysis and countermeasures of children's piano learning weariness.” (2) China Music Education Network: China music education network is a national music education resource and information website sponsored by the music education branch of the Chinese Education Association. It can provide necessary courseware, materials, and data support for music teaching in schools at all levels throughout the country and provide timely teaching and research information for the majority of music educators and researchers. (3) Improved association rule algorithm of China guzheng network: China guzheng network is a music education resource station in the guzheng professional field. It is divided into two parts: the “whole station home page” and the “TV channel home page.” “Home page” provides music scores and knowledge about guzheng music; “TV channel homepage” provides guzheng teaching video. (4) Hongxiao music education workstation: the station was founded by Zhao Hongxiao, a cucurbit flute player, and belongs to the personal music education resource website. The website is simple and colorful. It is mainly aimed at teachers and students and music lovers, providing them with a platform to exchange music teaching experience and learning experience.

Each line of data used represents a record and is stored in the form of file. The support used is 0.07, and there are eight nodes in the cluster.  Table 2 shows the data amount and time used for the test.

It can be seen from Figure 3 that when the data volume is 6000 records, the time difference between the Apriori algorithm based on the map improved association rule algorithm reduce framework and the classical Apriori algorithm is only more than 30 seconds. With the increase of the data volume, the gap is gradually narrowed. The proportion of the time spent processing data to the total running time increases, and the communication cost can be ignored. The following conclusions can be drawn. With the increase of data volume, the advantages over single machine are more obvious.

In this experiment, the acceleration ratio is taken as an important criterion.

Figures 4 and 5 show that when the number of nodes is less than or equal to 2, the consumption time gap is small. With the increase of the number of nodes, the acceleration ratio gap becomes larger and larger. It shows that when the number of nodes is greater than a certain number, the more nodes, the faster the processing speed and the higher the efficiency.

Compared with frequent itemsets, the algorithm for generating association rules is relatively simple. Generating association rules from frequent itemsets requires all its nonempty subsets first. As we can see, some of the attributes we are interested in are vacant, and the attribute values are missing. For example, learners did not take the final exam for some reason, resulting in the vacancy of total scores. For the attributes of these vacancies, data cleaning techniques can be used to fill them, for example, averaging, manually filling in vacancy values, or filling them with a specific character, because some attributes need to be discretized to use the decision tree method.

From Figure 6 improved association rule algorithm, it can be seen that the gap gradually increases with the increase of data volume.

Figure 7 displays the algorithm's acceleration ratio. The vertical axis displays the acceleration ratio, and the horizontal axis the number of nodes. The acceleration ratio is 1.31 for a node count of 2, 1.70 for a node count of 4, and 2.4 for a node count of 8. This indicates that the test data size is 1 m. It is evident that as the Hadoop cluster grows in size, so does the acceleration ratio for this technique. Common rule generation algorithms frequently experience issues like memory overflow and lengthy run times when dealing with big amounts of data. This section's rule generation algorithm, mapreducegenrules, can get around the previous approach. The algorithm's performance has greatly increased thanks to the use of a Hadoop cluster to process large amounts of data.

It can be found by comparing with the frequent 2-term set ({a, D}, {B, C}, {C, e}, {a, B}, {a, C}, and {C, D}) calculated by the traditional DHP algorithm. There are no itemsets {a, D}, {B, C}, {a, B}, and {C, D} in the frequent 2-term results of the new improved algorithm. In addition, the support of {a, D}, {a, B}, and {C, D} itemsets does not even meet the minimum support threshold of Apriori. The itemset {B, C} cannot be considered as a real frequent itemset because the items are not positively related. The new improved algorithm and the introduction of PCC threshold can not only reduce the size of candidate set but also ensure the quality of candidate set.

## 5. Conclusion

The construction of network music education resources in China has made great progress and gratifying achievements in recent years. However, due to the influence and restriction of various factors, there are still a series of problems in the construction of network music education resources, such as “the number of regional network music education resources sites is small, the coverage is small”; “the search function is not perfect and the efficiency is low”; “the construction of music courseware library is single and lacks the guidance of product awareness”; “the form of network music curriculum resources is single, the interaction is insufficient”; and “the navigation function design is insufficient.” Based on this, we should formulate the strategy of developing and integrating online music education resources on the basis of concrete research on the development trend of modern network information technology. These strategies generally include adopting rich hypertext and hypermedia methods to integrate and construct the knowledge system, teaching cases and material system of online music courses, promoting the optimal design of human-computer interaction, and helping teachers and students to create teaching “situations.” Provide a collaborative communication environment for music teaching, and build an effective mechanism for knowledge discovery and innovation. In the management of online music education resource database, the server operating system and database management system supporting the future “cloud computing” function are introduced to adapt to the future technological development trend.

## Figures and Tables

**Figure 1:** Basic operation mode of OOC.

**Figure 2:** DM flow chart of improved association rule algorithm.

**Figure 3:** Data comparison test of improved association rule algorithm.

**Figure 4:** Test diagram of different nodes of the improved association rule algorithm.

**Figure 5:** Test chart of speedup ratio of the improved association rule algorithm.

**Figure 6:** Comparison of running time.

**Figure 7:** Acceleration ratio test diagram.

**Table 1:** Simplified table of course evaluation mapping of improved association rule algorithm.

Course name	2013203561	2013203561	2013203561	2013203561	2013203561
100001	1	0	2	1	0
100002	2	0	5	1	2
100003	5	5	1	2	0
100004	4	4	0	6	5
100005	3	1	6	3	1
100006	2	3	2	3	3
100007	4	2	3	1	0

**Table 2:** Test data and time of improved association rule algorithm.

Number of records	6	120	250	500	1000	2000	2500	3200
MapReduce a priori test time	80	93	140	302	622	810	950	1200
Apriori test time	110	160	302	540	845	1523	2861	3210

## Data Availability

The data used to support the findings of this study are available from the corresponding author upon request.
